This article has been retracted.

# Metabonomic Study of the Effect of Dingkundan Intervention Comparing with Oral Contraceptives on Primary Dysmenorrhea Using the UPLC-MS Technique

**DOI:** 10.1155/2022/6708200

**Published:** 2022-08-17

**Authors:** Hong Cai, Yijing Zhang, Xiaoxia Ding, Shiyang Zhu, Xuesong Ding, Yan Deng, Xiao Ma, Jingwen Gan, Yanfang Wang, Aijun Sun

**Affiliations:** ^1^Affiliated Hangzhou First People's Hospital, Zhejiang University School of Medicine, Hangzhou, 310006 Zhejiang, China; ^2^National Clinical Research Center for Obstetrics & Gynecologic Diseases, Department of Obstetrics and Gynecology, Peking Union Medical College Hospital, Chinese Academy of Medical Sciences & Peking Union Medical College, Beijing, China

## Abstract

Primary dysmenorrhea (PD) is a prevalent problem in gynecologic clinics among adolescents and women of reproductive age. Several therapy modalities, including traditional Chinese medicine, are deemed adequate (TCM) and have been in practice for a long time. In China, Dingkundan (DKD), a multicomponent gynecological treatment, has been used to treat PD for centuries. However, the fundamental process remains poorly understood. Comparing plasma samples acquired from DKD-treated and oral contraceptive- (OC-) treated subjects, we performed an integrated plasma metabonomic analysis utilizing the UPLC-MS technology to study the therapeutic mechanisms of DKD in PD patients. Thirty possible biomarkers and metabolic pathways were discovered, primarily steroid hormone production, glycerophospholipid metabolism, and bile secretion. The results suggested that DKD may have therapeutic benefits for PD patients via modulation of various metabolic pathways. This study is envisaged to provide detailed metabolite information regarding the etiology of PD, an assessment of the efficacy of DKD, and a comparison of DKD and OC.

## 1. Introduction

PD (primary dysmenorrhea) is associated with painful uterine contracts incited due to endometrial perforation, starting several days before menstruation and ending for about 48 to 72 hours, where the pain is most prominently felt in the thigh muscles [1]. Primary dysmenorrhea (PD) is a painful uterine contraction caused by endometrial perforation. The pain associated with dysmenorrhea begins several days before the onset of menstruation and lasts between 48 and 72 hours, affecting the thighs and frequently being associated with cramping pain [1]. Dysmenorrhea is one of the most common problems among adolescent and adult ladies. Besides pain, it is accompanied by headache, lethargy, fatigue, hyperhidrosis, and muscle spasms. Dysmenorrhea prevalence has been found to be between 45 and 97% in the female population [2, 3]. Though the exact mechanism and manifestation of dysmenorrhea are still unknown, it has been suggested that prostaglandin syntheses, preferably E2 and F2, are major players in inducing ischemia and hypoxia, which then translate into uterine contraction and less blood flow to the affected areas [1, 4].

Dysmenorrhea is predominantly treated by the use of various drugs as well as different complementary medicines for a long time [5–7]. NSAIDs and OCs are the most frequently prescribed medicines, which hinder prostaglandins' production and subsequent release, thereby relieving pain. However, long-term use of NSAIDs is associated with various adverse effects, namely, nausea, vomiting, stomach, and duodenal ulcers owing to the nonselective nature of COX enzyme inhibition. In contrast, OC's excessive use may result in anorexia, asthma precipitation, and ace [8, 9].

The OC exerts its action by halting the ovulation stage during the menstrual cycle, reducing endometrial perforation, and enabling endometrial milieu during the early stages of the menstrual cycle, at the time when the prostaglandins are at their lowest level, thereby helping in alleviating the pain. Similarly, other ways of dealing with dysmenorrhea are also reported in the literature like exercising yoga, massaging the affected muscles, use of different supplements like vitamins and minerals, use of acupressure, use of acupuncture [1, 3, 6], and use of different herbal drugs like chamomile, ginger, and fennel [2, 10]. Nevertheless, neither NSAIDs nor natural plants can be the ultimate choice, owing to the former being prone to exacerbate digestive tract problems and the latter not readily available.

Dingkundan (DKD) is one of the most well-known traditional Chinese medicine (TCM) formulae that has demonstrated promising results for over three centuries. TCM is advocated with the advantage of the lesser extent of adverse effects associated with allopathic medicines. However, the mechanism has not been appropriately studied.

This study is aimed at investigating untargeted plasma metabonomic analysis to elucidate the therapeutic mechanism of DKD and compared the metabonomic profiles of DKD with hormonal therapy, one of the first-line management, to explore a better understanding of the difference.

## 2. Methods

### 2.1. Study Populations

A total of seventy-eight patients were recruited in a prospective, double-blind, multicenter, randomized controlled trial designed for primary dysmenorrhea treatment in China from June 2019 to December 2019. All participants enrolled reported a definitive history of primary dysmenorrhea. Patients were separated into two groups: OC treatment (group 1, *n* = 28) and DKD treatment (group 2, *n* = 50) for three months.

Inclusion criteria for this study include nonpregnant women aged between 16 and 35 years, regular menstruation (duration within 3–7 days, cycle within 21–35 days), ability to participate in the 3-month intervention study, and face-to-face follow-up interviews.

Written informed consent was provided to every participant, and the institutional review board approved the study at every medical center.

Patients with a history of secondary dysmenorrhea not limited to endometriosis, adenomyosis, and pelvic inflammatory disease; patients using medications containing female hormones or similar formulae to DKD prior to the study; patients addicted to alcohols and cigars; patients with unstable physical conditions; patients in the first year postpartum or lactating; patients with allergy to any pharmaceutical ingredients contained in OC and DKD; patients with a history or prone to have a thrombotic disease; patients with malignant disease; and patients with uterine endometrial abnormalities were excluded.

### 2.2. Plasma Sample Collection and Preparation

Blood samples were collected in fasting conditions before and after treatment, were subjected to centrifugation to separate plasma, and were frozen immediately at −80°C. Before use, all samples were thawed at 4°C in an ice bath, and accurately measured, 100 *μ*L was taken and added into 400 *μ*L of methanol: water mixture (4 : 1 *v*/*v*) to extract the metabolites. All samples were then kept at −20°C and homogenized using a high-throughput tissue crusher (Wonbio-96c, Shanghai Wanbo Biotechnology Co. Ltd.) at a frequency of 50 Hz for 6 minutes, followed by vortexing for 30 seconds, and subjected to ultrasound treatment at 40 kHz for 30 minutes at 5°C. The samples were then allowed to stand for 30 minutes at −20°C for protein precipitation, followed by centrifuging all samples at 13000 g for 15 minutes at 4°C. The supernatants were carefully separated and collected for subsequent analysis.

### 2.3. UPLC-MS Analysis

All samples were subjected to UPLC-MS analysis using the ExionLC™ AD system (AB Sciex, USA). The column used was ACQUITY UPLC BEH C18 (dimensions 100 mm × 2.1 mm, 1.7 *μ*m; Waters Milford, USA). The UPLC was coupled with a quadrupole-time-of-flight mass spectrometer (Triple TOFTM5600+, AB Sciex, USA) and an electrospray ionization (ESI) source operating in both the positive mode and the negative mode. The analysis was performed over a mass range of 50–1000 m/z.

### 2.4. Data Interpretation

Following running each sample on the UPLC-MS system, the data obtained was transported to Progenesis (QI 2.3, Nonlinear Dynamics, Waters, USA) for peak detection and alignment. Different metabolites were detected, and at least 80% in any set of samples was considered retained. The actual mass of each metabolite was used for identification purposes of the mass spectra of metabolites. Furthermore, two different biochemical databases (Human Metabolome http://www.hmdb.ca/ and METLIN database https://metlin.scripps.edu/) were consulted for identifying MS/MS fragment spectra and for distinguishing isotope ratio differences.

## 3. Statistical Analysis

All obtained data were statistically analyzed employing different tests like multivariant analysis (ropls, version 1.6.2) and R package from the Bioconductor on Majorbio Cloud Platform. The panoramic view of metabolites was tested using principal component analysis (PCA), and overall metabolite changes between groups were analyzed using orthogonal partial least square discriminate analysis (OPLS-DA) with variable importance in the projection (VIP). The model parameters, i.e., R2 and Q2, were calculated to provide information for interpretability and predictability. The *P* values were determined using paired Student's *t*-test, and the significance level was set to *P* < 0.05.

## 4. Results

### 4.1. Clinical Characteristics and Outcomes

Clinical characteristics of participants in this study are listed in Table 1. There was no statistical difference between the DKD and OC groups in parameters including the year of age, procreated ratio, menstruation information, age of menarche, menstrual bleeding duration, and menstrual cycle length. Both cohorts collected visual analogue scale (VAS) scores before and after treatment. Results showed distinguish relief in VAS scores after treatment in both groups compared to baseline data (*P* < 0.01). Participants in OC groups reported lower VAS scores after treatment compared to those in DKD groups (*P* < 0.01), but there was no statistical difference in the overall effective rate between DKD and OC groups (*P* = 0.06).

### 4.2. OPLS-DA

Pairwise comparisons between the two groups revealed DKD and OC-related serum metabolites. Partial separation was shown in the OPLS-DA model with R2Y (cum) = 0.667 and Q2 (cum) = 0.349 (Figure 1(a)). The S-plot and VIP value showed the metabolic effect of DKD (Figure 1(b)). A total of 104 specific metabolites were distinguished from two groups. Only metabolic compounds that met the criteria of both projection (VIP) value > 2.5 and *P* value < 0.05 were identified as potentially different (Table 2). Most of these differential metabolites were lipids and lipid-like compounds, including elevated levels of glycinoeclepin, taurodeoxycholic acid, bromo fatty acid, dihydroxycholest, traumatic acid, etc. and decreased levels of lysophospholipid, lipopolysaccharide, bile acid, cortisol, phosphatidylcholine, etc.

### 4.3. Hierarchical Cluster Analysis

Hierarchical cluster analysis is commonly used for quantitative classification. Data were visualized by an HCA heat map (Figure 2). The result indicated that 78 tested samples (containing 50 DKD and 28 OC samples) could be divided into ten categories based on their chemical composition differences. The heat map showed that the steroid hormone-associated content (tocotrienol, androsterone sulfate, and estrone glucuronide) was at higher levels in DKD than in OC, while the contents of phosphatidylcholine, lysophospholipid, and cortisol were at lower levels accordingly.

### 4.4. Pathway Enrichment Analysis

Detailed impacts of DKD and OC-related alterations in metabolic networks were shown in Figure 3. A pathway impact > 0.05 and log (*P*) > 20 were considered the most important. Twenty metabolic pathways were identified, including the steroid hormone biosynthesis, bile secretion, glycerophospholipid metabolism, alpha-linolenic acid metabolism, choline metabolism in cancer, and aldosterone-regulated sodium reabsorption.

Eight metabolites showed to be enriched in KEGG pathway analysis. The serum levels of HMDB0007884 (PC(14:0/20:4(8Z,11Z,14Z,17Z))), HMDB0000564 (PC(16:0/16:0)), and HMDB0000063 (cortisol) were significantly decreased in the DKD group compared with the OC group (all *P* < 0.01), while OC treatment elevated the concentrations of HMDB0000145 (estrone), HMDB0000933 (traumatic acid), HMDB0010318 (pregnanediol-3-glucuronide), HMDB0001032 (dehydroepiandrosterone sulfate), and HMDB0004483 (estrone glucuronide) (Figure 4).

## 5. Discussion

Aiming at investigating the serum metabolic profile of primary dysmenorrhea after DKD treatment, we performed the clinical study using an LC-MS-based metabolomics technique. Furthermore, DKD treatment was compared with oral contraceptives, considered first-line management [10]. The randomized, double-blind trial setting assesses the efficacy of DKD in primary dysmenorrhea. Results showed similar therapeutic outcomes between the two groups that indicated that DKD could be an alternative option for those PD patients who do not want or have contraindications to hormone medicine.

Further analysis revealed partial separation between DKD and OC groups based on metabolic profiling. Most of the differential metabolites were lipids and lipid-like compounds. Several metabolic pathways were involved, including the steroid hormone biosynthesis, bile secretion, glycerophospholipid metabolism, alpha-linolenic acid metabolism, choline metabolism in cancer, and aldosterone-regulated sodium reabsorption. Among these pathways, steroid hormone biosynthesis and bile secretion were impacted most. It is widely accepted that oral contraceptives could manage menstrual pain by suppressing ovulation and endometrial proliferation to block the production of prostaglandins, which also involve alternation of steroid hormone dynamics. At the same time, DKD may contribute to pain relieving through nonsteroid hormone metabolic pathways. KEGG enrichment analysis showed that DKD decreased PC(16:0/16), cortisol, and PC(14:0/20:4(8Z,11Z,14Z,17Z)) in serum levels compared with hormonal therapy, while elevating estrone, estrone glucuronide, traumatic acid, pregnanediol-3-glucuronide, and dehydroepiandrosterone sulfate levels.

PC (16:0/16) is metabolized in PC synthesis and the glycerophospholipid metabolism pathway, and disturbance of the latter is associated with depression. Recent studies revealed that serum levels of PC (16:0/16) were elevated in antenatal depression and showed a positive trending correlation with depression scores [11–13]. Abundant evidence has uncovered psychological risk factors associated with PD, including depression and anxiety, and psychotherapy interventions are considered effective in PD accordingly [14, 15]. Our results also showed remarkably lower PC(16:0/16) serum levels in DKD profiles, which indicated that regulation of PC-involved metabolic pathways might be employed as an antidepression method.

Cortisol is regarded as downstream production of the hypothalamic-pituitary-adrenal (HPA) axis and reflects the activation of the central nervous system, which is also the primary pain response system. Patients complaining of chronic pain often present with hypercortisolism, and nonpharmacological therapeutics, cognitive behavioral therapy, and exercise are regarded as promising options in treating centralized pain with serum cortisol level downregulation observed as well [16, 17]. PD is also identified as a central oversensitivity syndrome characterized by pain hypersensitivity without physical organ injury or a nervous system lesion with both peripheral and central hypersensitivity to pain [18]. Our data revealed significant downregulated cortisol levels in the DKD group compared to OC treatment, hinting that DKD may positively affect pain by improving HPA axis regulation.

Estrone, estrone glucuronide, and pregnanediol-3-glucuronide are hormonal steroids and reflect longer-term levels of E2 and P4 in circulation. Oral contraceptives could suppress the concentrations of the abovementioned metabolites by ovulation suppression.

DKD is one of the most widely used Chinese traditional medicines. It helps alleviate pain, regulate menstrual function, and nourish ovarian function. The components of DKD include red ginseng, saffron, *cornu-cervi*, *Radix rehmanniae preparata*, *Radix paeoniae alba*, *Angelica sinensis*, *Scutellaria baicalensis*, *Cyperi rhizoma*, *Rhizoma chuanxiong*, motherwort fruit, and *Rhizoma corydalis*. Among these components, red ginseng, *Rhizoma chuanxiong*, saffron, and *Rhizoma corydalis* were the main ingredients for pain relief. Lee et al. suggested that Rb1, the most representative ginsenoside, inhibits inflammatory response and achieves antinociceptive effects by downregulating the activation of L4-L5 spinal cord microglia and astrocytes and potentially through the estrogen receptor [19]. *Rhizoma chuanxiong* (RCX) is another popular TCM herb that possesses efficacy in alleviating pain. Pharmacological studies have demonstrated bioactivities of RCX, including uterus contraction regulatory activity, antimigraine activity, neuroprotective activity, cardioprotective activity by blocking calcium channels, and antivascular smooth muscle proliferation antioxidant, antiplatelet aggregation, and antithrombosis, and anti-inflammation effects [20]. Saffron has been a folk remedy for pain, cramps, and depressive disorder for a long time. Studies showed that crocin might be the main active component with various pharmacological effects. Clinical studies and animal models have shown that saffron makes an effort on pain relief such as PD, osteoarthritis, and neuropathic pain [21–25]. According to Khan et al., saffron may not act through central mechanisms [26]. Other studies suggested that saffron may retard NF-*κ*B activation through JNK signaling pathway inhibition and repress IL-6 expression and oxidative stress in turn as well [27]. *Rhizoma corydalis* (RC) is another vital compound in ancient China's classical pain relief formula. Recent studies have discovered that RC has a noticeable antinociceptive effect on the central dopaminergic system. A remarkable effect of antidepression and sedative activity is also reported in patients treated with RC in different diseases [28, 29].

## 6. Conclusion

This work was carried out to investigate the different roles and possible mechanisms of DKD compared to OC for PD by a UPLC-MS-based metabolomics method. We identified 104 compounds in serum with significant metabolic changes. The metabolic pathway analysis showed that the different mechanism was mainly involved in steroid hormone biosynthesis, bile secretion, glycerophospholipid metabolism, alpha-linolenic acid metabolism, choline metabolism in cancer, and aldosterone-regulated sodium reabsorption. Interpretation results showed downregulation of PC activity (16:0/16:0) and cortisol. In contrast, upregulation of the activity of traumatic acid may be responsible for the different effects of DKD compared with OC. Further studies emerged to investigate DKD treatment on PD with more functionally validated metabolite changes. This study also reveals that the LC-MS-based untargeted metabolomics technique may be a promising tool for exploring the mechanism of TCM formulas.

## Figures and Tables

**Figure 1:** Score plot and S-plot for the OPLS-DA model between DKD and OC groups.

**Figure 2:** Heatmap of hierarchical clustering for the DKD group and OC group. The abscissa represents different experimental sets, the ordinate represents the differential metabolites clustered, and the color represents the relative content of metabolites in the corresponding sample, red for higher and blue for lower contents.

**Figure 3:** KEGG pathway enrichment. (a) KEGG pathway enrichment bubble plot. (b) KEGG pathway classification chart.

**Figure 4:** Metabolites enriched in the KEGG pathway. Relative expressions of HMDB0007884 (PC(14:0/20:4(8Z,11Z,14Z,17Z))), HMDB0000564 (PC(16:0/16)), HMDB0000063 (cortisol), HMDB0000145 (estrone), HMDB0000933 (traumatic acid), HMDB0010318 (pregnanediol-3-glucuronide), HMDB0001032 (dehydroepiandrosterone sulfate), and HMDB0004483 (estrone glucuronide) in serum with DKD and OC treatment. ^∗∗^*P* < 0.01, ^∗^*P* < 0.05.

**Table 1:** Clinical characteristics and treatment results of participants in this study.

	DKD cohort (*n* = 50)	COC cohort (*n* = 28)	*P* value
Age (years)	24.63 ± 4.11	26.24 ± 4.49	0.38
Age of menarche (years)	12.79 ± 1.12	12.85 ± 1.23	0.85
Menstrual cycle length (days)	29.50 ± 4.58	30.41 ± 2.94	0.25
Menstrual bleeding duration (days)	6.00 ± 1.12	6.09 ± 1.38	0.39
Procreated rate (%)	6.00	17.86	0.23
VAS before treatment	3.82 ± 1.78	4.56 ± 2.34	0.36
VAS after treatment	2.93 ± 0.27^∗^	1.78 ± 0.28^#^	<0.01
Pain relief response			
Marked moderate (*n*)	29	22	
No relief (*n*)	21	6	
Overall effective rate (%)	58.0	78.6	0.06

^∗^Compared with VAS before treatment, *P* < 0.01; ^#^compared with VAS before treatment, *P* < 0.01.

**Table 2:** Statistical analysis of differential metabolites from two groups.

Metabolite	VIP_pred_OPLS-DA	FC(DKD vs. OC)	*P* value
Glycinoeclepin A	4.52	1.24	<0.001
9-Hydroxy-10-O-D-glucuronoside-12Z-octadecenoate	4.10	0.74	0.004
N,N′-Diacetylchitobiose	3.96	1.15	0.008
Tauroursodeoxycholic acid	3.79	0.81	<0.001
12-Bromo-dodecanoic acid	3.52	1.07	<0.001
3′-N′-Acetylfusarochromanone	3.52	1.07	<0.001
(25R)-3Beta,4beta-dihydroxycholest-5-en-26-oate(1-)	3.39	1.12	<0.001
Ferulic acid	3.39	0.84	0.001
N-(1-Deoxy-1-fructosyl)tryptophan	3.33	1.08	0.007
Taurodeoxycholic acid	3.15	0.91	0.004
L-N-(1H-Indol-3-ylacetyl)glutamic acid	3.10	1.06	0.001
1-Phenyl-1,3-eicosanedione	2.92	1.06	<0.001
Fluvoxamino acid	2.90	1.04	0.003
2-Amino-5-phenylpyridine	2.90	1.05	<0.001
Cortisol	2.88	0.95	<0.001
Traumatic acid	2.84	1.10	0.005
LysoPE(0:0/15:0)	2.83	0.88	0.001
Thiomorpholine 3-carboxylate	2.81	1.13	0.020
Taurochenodeoxycholate-7-sulfate	2.79	0.94	0.001
Piperine	2.77	1.15	0.009
4-Cholesten-7alpha,12alpha,24-triol-3-one	2.73	1.05	<0.001
Cytochalasin Ppho	2.72	0.80	0.042
3′-Ketolactose	2.71	1.05	0.005
16-Bromo-9E-hexadecenoic acid	2.71	1.03	0.003
7′-Carboxy-gamma-tocotrienol	2.68	0.94	<0.001
Cis-5-Tetradecenoylcarnitine	2.66	1.11	0.019
15-Octadecene-9,11,13-triynoic acid	2.62	1.05	0.014
Inosine	2.61	0.93	0.041
(±)-Rollipyrrole	2.58	1.06	<0.001
Neomenthol-glucuronide	2.56	1.08	0.012

## Data Availability

The datasets during and/or analyzed during the current study are available from the corresponding author upon reasonable request.

## References

[1] Xu Y., Zhao W., Li T. (2017). Effects of acupoint-stimulation for the treatment of primary dysmenorrhoea compared with NSAIDs: a systematic review and meta-analysis of 19 RCTs. *BMC Complementary and Alternative Medicine*.

[2] Kim K. I., Nam H. J., Kim M., Lee J., Kim K. (2017). Effects of herbal medicine for dysmenorrhea treatment on accompanied acne vulgaris: a study protocol for a randomized controlled trial. *BMC Complementary and Alternative Medicine*.

[3] Lee H., Choi T. Y., Myung C. S., Lee M. S. (2016). Herbal medicine Shaofu Zhuyu decoction for primary dysmenorrhea: a systematic review protocol. *Systematic reviews*.

[4] Ghafourian M., Band N. A., Pour A. F., Kooti W., Rad M. F., Badiee M. (2015). The role of CD16+, CD56+, NK (CD16+/CD56+) and B CD20+ cells in the outcome of pregnancy in women with recurrent spontaneous abortion. *International Journal of Women's Health and Reproduction Sciences*.

[5] Chao M. T., Wade C. M., Abercrombie P. D., Gomolak D. (2014). An innovative acupuncture treatment for primary dysmenorrhea: a randomized, crossover pilot study. *Alternative Therapies in Health and Medicine*.

[6] Hosseinlou A., Alinejad V., Alinejad M., Aghakhani N. (2014). The effects of fish oil capsules and vitamin B1 tablets on duration and severity of dysmenorrhea in students of high school in Urmia-Iran. *Global Journal of Health Sciences*.

[7] Kooti W., Mansouri E., Ghasemiboroon M., Harizi M., Ashtary-Larky D., Afrisham R. (2014). The effects of Hydroalcoholic extract of Apium graveolens leaf on the number of sexual cells and testicular structure in rat. *Jundishapur Journal of Natural Pharmaceutical Products*.

[8] Navvabi Rigi S., Kermansaravi F., Navidian A. (2012). Comparing the analgesic effect of heat patch containing iron chip and ibuprofen for primary dysmenorrhea: a randomized controlled trial. *BMC Women’s Health*.

[9] Rahnama P., Montazeri A., Huseini H. F., Kianbakht S., Naseri M. (2012). Effect of Zingiber officinale R. rhizomes (ginger) on pain relief in primary dysmenorrhea: a placebo randomized trial. *BMC Complementary and Alternative Medicine*.

[10] Kho K. A., Shields J. K. (2020). Diagnosis and management of primary dysmenorrhea. *Journal of the American Medical Association*.

[11] Mao Q., Tian T., Chen J., Guo X., Zhang X., Zou T. (2021). Serum metabolic profiling of late-pregnant women with antenatal depressive symptoms. *Frontiers in Psychiatry*.

[12] Wu Z., Zhao P., Long Z. (2019). Biomarker screening for antenatal depression in women who underwent caesarean section: a matched observational study with plasma lipidomics. *BMC Psychiatry*.

[13] Zhao S., Wu W., Kang R., Wang X. (2021). Significant increase in depression in women with primary dysmenorrhea: a systematic review and cumulative analysis. *Frontiers in Psychiatry*.

[14] Bajalan Z., Moafi F., MoradiBaglooei M., Alimoradi Z. (2019). Mental health and primary dysmenorrhea: a systematic review. *Journal of Psychosomatic Obstetrics and Gynaecology*.

[15] Gagua T., Tkeshelashvili B., Gagua D., McHedlishvili N. (2013). Assessment of anxiety and depression in adolescents with primary dysmenorrhea: a case-control study. *Journal of Pediatric and Adolescent Gynecology*.

[16] Eller-Smith O. C., Nicol A. L., Christianson J. A. (2018). Potential mechanisms underlying centralized pain and emerging therapeutic interventions. *Frontiers in Cellular Neuroscience*.

[17] Zheng H., Liu Y., Li W. (2006). Beneficial effects of exercise and its molecular mechanisms on depression in rats. *Behavioural Brain Research*.

[18] Iacovides S., Avidon I., Baker F. C. (2015). What we know about primary dysmenorrhea today: a critical review. *Human Reproduction Update*.

[19] Lee J. Y., Choi H. Y., Park C. S., Kim D. H., Yune T. Y. (2021). Total saponin extract, ginsenoside Rb1, and compound K alleviate peripheral and central neuropathic pain through estrogen receptors on rats. *Phytotherapy Research*.

[20] Pu Z. H., Dai M., Xiong L., Peng C. (2020). Total alkaloids from the rhizomes of Ligusticum striatum: a review of chemical analysis and pharmacological activities. *Natural Product Research*.

[21] Sacks D., Baxter B., BCV C. (2018). Multisociety consensus quality improvement revised consensus statement for endovascular therapy of acute ischemic stroke. *International journal of stroke*.

[22] Mohammad N. S., Nazli R., Zafar H., Fatima S. (2022). Effects of lipid based multiple micronutrients supplement on the birth outcome of underweight pre-eclamptic women: a randomized clinical trial. *Pakistan Journal of Medical Sciences*.

[23] Hausenblas H. A., Saha D., Dubyak P. J., Anton S. D. (2013). Saffron (Crocus sativus L.) and major depressive disorder: a meta-analysis of randomized clinical trials.

[24] Kell G., Rao A., Beccaria G., Clayton P., Inarejos-García A. M., Prodanov M. (2017). Affron® a novel saffron extract (Crocus sativus L.) improves mood in healthy adults over 4 weeks in a double-blind, parallel, randomized, placebo-controlled clinical trial. *Complementary Therapies in Medicine*.

[25] Nahid K., Fariborz M., Ataolah G., Solokian S. (2009). The effect of an Iranian herbal drug on primary dysmenorrhea: a clinical controlled trial. *Journal of Midwifery & Women’s Health*.

[26] Khan A., Muhamad N. A., Ismail H. (2020). Potential nutraceutical benefits of in vivo grown saffron (Crocus sativus L.) as analgesic, anti-inflammatory, anticoagulant, and antidepressant in mice. *Plants*.

[27] Lei M., Guo C., Hua L. (2017). Crocin attenuates joint pain and muscle dysfunction in osteoarthritis rat. *Inflammation*.

[28] Pao L. H., Lu S. W., Sun G. G., Chiou S. H., Ma K. H. (2012). Three Chinese herbal medicines promote neuroproliferation in vitro, and reverse the effects of chronic mild stress on behavior, the HPA axis, and proliferation of hippocampal precursor cell in vivo. *Journal of Ethnopharmacology*.

[29] Wu H., Wang P., Liu M. (2015). A 1H-NMR-based metabonomic study on the anti-depressive effect of the total alkaloid of corydalis rhizoma. *Molecules*.

